# Bleomycin induces epithelial-to-mesenchymal transition via bFGF/PI3K/ESRP1 signaling in pulmonary fibrosis

**DOI:** 10.1042/BSR20190756

**Published:** 2020-01-14

**Authors:** Chang-Mei Weng, Qing Li, Kui-Jun Chen, Cheng-Xiong Xu, Meng-Sheng Deng, Tao Li, Dong-Dong Zhang, Zhao-Xia Duan, Zhi-Qiang Chen, Guan-Hua Li, Jing Chen, Jian-Min Wang

**Affiliations:** 1 Research Institute of Surgery, Daping Hospital, Army Medical University, Chongqing 400042, People’s Republic of China; 2 State Key Laboratory of Trauma Burn and Combined Injury, Chongqing 400042, People’s Republic of China; 3 Cancer Center, Daping Hospital, Army Medical University, Chongqing 400042, People’s Republic of China; 4 Joint Surgery Center, Southwest Hospital, Army Medical University, Chongqing 400038, China

**Keywords:** bFGF, Bleomycin, EMT, PI3K/Akt Signaling, Pulmonary Fibrosis

## Abstract

Idiopathic pulmonary fibrosis (IPF) is a fatal and chronic disease with a high rate of infection and mortality; however, its etiology and pathogenesis remain unclear. Studies have revealed that epithelial–mesenchymal transition (EMT) is a crucial cellular event in IPF. Here, we identified that the pulmonary fibrosis inducer bleomycin simultaneously increased the expression of bFGF and TGF-β1 and inhibited epithelial-specific regulatory protein (ESRP1) expression *in vivo* and *in vitro*. In addition, *in vitro* experiments showed that bFGF and TGF-β1 down-regulated the expression of ESRP1 and that silencing ESRP1 promoted EMT in A549 cells. Notably, we determined that bFGF activates PI3K/Akt signaling, and treatment with the PI3K/Akt inhibitor LY294002 inhibited bleomycin-induced cell morphology changes and EMT. In addition, the effects of LY294002 on bleomycin-induced EMT were inhibited by ESRP1 silencing in A549 cells. Taken together, these findings suggest that bleomycin induced EMT through down-regulating ESRP1 by simultaneously increasing bFGF and TGF-β1 in pulmonary fibrosis. Additionally, our findings indicated that bFGF inhibits ESRP1 by activating PI3K/Akt signaling.

## Introduction

Pulmonary fibrosis (PF) is the proliferation of lung fibroblasts and the accumulation of a large number of extracellular matrix components, resulting in distortion of alveolar architecture and interstitial pneumonia, even leading to progressive loss of lung function with breathing difficulty, respiratory deterioration and other interstitial lung diseases. It has been called a ‘tumor-like disease’ due to its higher morbidity and mortality than most tumors [1]. Epithelial–mesenchymal transition (EMT) is a critical event in pathophysiological progression, such as fibrosis and cancer progression. In pulmonary fibrosis, oval alveolar epithelial cells lose their polarity and specialized junction structures, gradually convert to elongated fusiform mesenchyme cells and resulting in the down-regulation of epithelial markers (E-cadherin) and the up-regulation of mesenchymal markers (N-cadherin, Vimentin, Fibronectin, α-SMA). Then, pulmonary calculi, even lung carcinoma, can develop without any intervention [2,3]. The progression and definite mechanism of EMT have been studied by researchers in recent decades, and various studies have suggested that targeting EMT will become a promising strategy for disease treatment [4].

Fibroblast growth factor receptors (FGFRs) are receptors of tyrosine kinases, which are expressed by tissue-specific alternative splicing in epithelial IIIb or mesenchymal IIIc isoforms. In appropriate specific alternative splicing of FGFRs is caused due to ordered expression of IIIb or IIIc isoforms and then lead to an imbalance of EMT [5]. Splicing regulatory proteins, specifically, epithelial-specific regulatory proteins (ESRPs) expressed in epithelial cells, play a pivotal role in the splicing procedure of FGFR2, which is related to the alternative splicing of FGFR2 IIIb and IIIc, further to achieve epithelial and mesenchymal isoforms, respectively [6]. A wealth of evidence strongly indicates that the elaborate programs of ESRP-regulated splicing events and coordinated biological functions are essential for epithelial cell function and other normal development. It is noteworthy that ESRP targets are assembled for genes/proteins involved in epithelial-cell properties such as cell–cell junctions, cell proliferation and differentiation, cell motility and pathways involved in EMT [7–9].

EMT is triggered and modulated by many signaling pathways, including PI3K/Akt (phosphatidylinositol 3 kinase), MAPK/Erk1/2, Smad2/3, Ras etc*.* These pathways are usually initiated by different cytokines, such as the TGF-β superfamily, fibroblast growth factor (FGF), epidermal growth factor (EGF) and integrins. Basic fibroblast growth factor (bFGF) belongs to the fibroblast growth factor family, which consists of 18 FGFs and 4 FGF receptors [10]. Earlier studies suggested that bFGF plays a protective role during cell death in animal models, including models of retinal damage [11,12]. In addition, recent investigations have indicated that bFGF is involved in wound healing and improves or reduces scar formation during the wound healing process [13]. Moreover, bFGF acts as a potent mitogen that stimulates the proliferation, differentiation and migration of mesenchymal cells [14]. In addition, in both hepatocellular carcinoma (HCC) and prostate cancer cells, bFGF was shown to induce epithelial–mesenchymal transition through the AKT/GSK-3β/Snail signaling pathway [15,16]. Although it has been reported that bFGF can induce EMT, the definite process remains to be elucidated. The probable mechanism was that phosphorylation of the pathways (pAKT/AKT/GSK-3β or MAPK/ERK) can be activated by bFGF, directly or indirectly.

Transforming growth factor (TGF-β) family members are multifunctional cytokines that are pivotal regulators of normal epithelial cell proliferation, differentiation and apoptosis, and the TGF-β/Smad2/3 pathway is widely recognized in EMT. Numerous studies have reported that TGF-β has been implicated as a ‘master switch’ in the induction of EMT. Increased expression of mesenchymal cell markers (Vimentin, α-SMA etc.) and decreased expression of epithelial cell markers (E-cadherin and cytokeratin) were found in TGF-β1-treated alveolar epithelial cells, A549 cells and bronchial epithelial cells [17–19]. In addition to its effect on the activation of Smad2/3, TGF-β also participates in other non-Smad signaling pathways to induce EMT, such as PI3K/Akt, ERK1/2 and MAPK [20,21], and can also alter cell behavior independently by stimulating nonreceptor protein tyrosine kinases, small GTP-binding proteins and MAP kinases [22,23].

The chemotherapeutic antibiotic-bleomycin (BLM) is widely used as an inducer of pulmonary fibrosis in animal models, and pro-inflammatory cytokines, pro-fibrotic proteins and fibrotic events were found in the lungs of mice that underwent intratracheal instillation of bleomycin [24]. Similar effects were validated *in vitro* experiments, and EMT characteristics were detected in bleomycin-treated A549 cells [25]. In this article, we investigate the role of ESRP1, TGF-β1 and bFGF in bleomycin-induced EMT and explore the underlying mechanisms of ESRP1 in TGF-β1 and bFGF-induced EMT. We have shown that significant differences in the expression of ESRP1, TGF-β1 and bFGF were indicated in bleomycin-induced pulmonary fibrosis, and apparent EMT signs were detected in siESRP1 cells that were treated with TGF-β1, bFGF and bleomycin. All results illustrated that the ESRP1 and bFGF play vital roles in bleomycin-induced EMT in A549 cells.

## Materials and methods

### Reagents and antibodies

Bleomycin (BLM) was obtained from Nippon Kayaku (Tokyo, Japan). TGF-β1 and primary antibodies against α-SMA (rabbit polyclonal) were purchased from Proteintech (Chicago, U.S.A.). The PI3K inhibitor LY294002 was obtained from Selleckchem (Houston, U.S.A.). Primary antibody against ESRP1 (rabbit polyclonal) was obtained from Sigma (Missouri, U.S.A.). E-cadherin (rabbit monoclonal), Vimentin (mouse monoclonal), bFGF (rabbit polyclonal), TGF-β1 (rabbit monoclonal), β-actin (mouse monoclonal) antibodies, horseradish peroxidase (HRP)-conjugated secondary antibodies, fluorescence secondary antibodies, ELISA kits, and recombinant human bFGF were all purchased from Abcam (Cambridge, U.K.). Primary antibodies against pAkt and Akt were obtained from Cell Signaling Technology (Boston, U.S.A.). DAPI, transfection reagent Lipofectamine 2000 and total RNA Reagent Trizol were purchased from Life Technologies (New York, U.S.A.). All histological and immunohistochemical reagents were purchased from Zhong-shan-Jin-qiao Biotechnology (Beijing, China). RNA interference sequences were obtained from RiboBio (Guangzhou, China). The PrimeScript®RT Reagent Kit with gDNA Eraser was a product of TaKaRa (Beijing, China). Quantitative real-time PCR kits (iTaq™ Universal SYBR® Green Supermix) were purchased from Bio-Rad (California, U.S.A.). Other chemical reagents were obtained from Sangon Biotech (Shanghai, China).

### Animal experiment

The animal experiments were performed in accordance with the guidelines and regulations of the Ethics Committee for Animal Experiments. Kunming mice (male, 27 ± 2 g, 4–6 weeks) were used to establish the model of lung fibrosis and were purchased from the animal center of Daping Hospital (Chongqing, China). All mice were maintained specific pathogen-free (SPF) conditions with free access to water and laboratory rodent food. Lung fibrosis was induced by bleomycin in mice as described as previously [26]. Briefly, following anesthesia with 0.1% pentobarbital, mice received slow intratracheal injection with 6 mg/kg of bleomycin dissolved in saline, while control mice received saline only. The treated mice were recovered and observed for 4 weeks and then sacrificed, and mouse lungs were obtained for histopathologic analysis.

### Histology

The lungs of mice were fixed in 4% (w/v) phosphate-buffered paraformaldehyde for 48 to 72 h, dehydrated, transparentized and embedded in paraffin. Lung tissues were cut into 3–5 μm sections that were stained with hematoxylin–eosin (H&E) for structured observation or with Masson’s trichrome stain for the detection of collagen distribution or were subjected to immunohistochemistry analysis.

### Immunohistochemistry analysis

Immunohistochemistry staining for the detection of ESRP1, TGF-β1 and bFGF *in vivo* was performed as the instruction manual. In brief, the slides were cleared of paraffin and subjected to antigen retrieval. Then, endogenous peroxidase activity was quenched with an endogenous peroxidase blocker, and the primary antibodies were employed (rabbit anti-TGF-β1, rabbit anti-FGF-2 and rabbit anti-ESRP1) at 4°C overnight. The secondary antibodies incubated were horseradish peroxidase-conjugated goat anti-rabbit/IgG, and immunoreactive proteins were detected using an Olympus microscope BX50 (Olympus BX50, Japan).

### Cell culture

The cell line A549 was purchased from the Shanghai Institute of Cell Biology. Cells were cultured in DMEM-F12 medium (Gibco-BRL, CA, U.S.A.) supplemented with 10% fetal bovine serum (Gibco-BRL), 100 μg/ml penicillin and 100 μg/ml streptomycin (Invitrogen) in an incubator with 5% CO_2_ at 37°C.

### ELISA

The measurements of TGF-β1 and bFGF were obtained as follows. The cell supernatant of A549 cells treated with 5 ng/ml TGF-β1 or 20 ng/ml bFGF for 48 h was collected, and a standard curve line was determined, and other steps were executed according to the instructions.

### RNA interference

siRNAs targeting the human ESRP1 are designed by Guangzhou RiboBio (Guangzhou, China), and target sites sequences are as below: ESRP1-001: GCACGAAGTGCTAGTTAGA, ESRP1-002: GCAAGATGGAACTTATTGA, ESRP1-003: GGGTTCACATGGTTTTGAA. RNA interference was determined as described in the instruction manual. A549 cells (2 × 10^5^ cells per well) were seeded in six-well plates, cultured for 24 h and then transfected with 50 nmol siRNA mixed with Lipofectamine 2000 reagent (Invitrogen) in serum-free medium according to the manufacturer’s instructions. The medium was changed to complete culture medium after 4 h. After another 24 h of incubation in a 37°C CO_2_ incubator, the cells were harvested for total RNA and total protein or treated with TGF-β1, bFGF, or bleomycin for other experiments.

### Isolation of RNA and reverse transcription-polymerase chain reaction (RT-PCR)

A549 cells were seeded at 0.7 × 10^5^ cells per well in six-well plates, and the medium was replaced with 2 ml of serum-free medium. Inhibitor LY294002 was added for pretreatment for 1 h before incubation with 5 ng/ml TGF-β1, 20 ng/ml bFGF or 20 µg/ml bleomycin for 48 h and then collected for subsequent experiments. Total RNA was extracted from the cells with Trizol and reverse transcribed with PrimeScript®RT Reagent Kit according to the manufacturer’s instructions.

### Quantitative real-time PCR

cDNA was subjected to 10 μl real-time PCRs carried out in an iCycler thermal cycler using SYBR Green Supermix with gene-specific primers (Invitrogen) (Table 1). The primers were designed from sequences available on GenBank (NIH genetic sequence database). After normalizing to the GAPDH and β-actin genes, the expression levels for each target gene were calculated using the comparative threshold cycle (*C*_T_) method. Data are presented as the fold change relative to the control using the 2^−ΔΔ*C*^_t_ method.

**Table 1:** Primers used in this study (Invitrogen)

Gene name	Forward primer (5′→3′)	Reverse primer (5′→3′)	Product size	Accession number
ESRP1	ACCGAGACCTAGCACTAC	ACTGGGCTACCTCATTGG	123 bp	XM_005250991.3
E-cadherin	TGCCCAGAAAATGAAAAAGG	GTGTATGTGGCAATGCGTTC	160 bp	XM_011523489.1
Vimentin	GAGAACTTTGCCGTTGAAGC	GCTTCCTGTAGGTGGCAATC	123 bp	XM_011519649.1
GAPDH	TCGACAGTCAGCCGCATCTTCTTT	GCCCAATACGACCAAATCCGTTGA	196 bp	NM_002046.3
β-actin	CATGTACGTTGCTATCCAGGC	CTCCTTAATGTCACGCACGAT	207 bp	NM_001100.3

### Total protein extract for Western blotting analysis

A549 cells were seeded in six-well plates (approximately 0.7 × 10^5^ cells per well). When cells were spread in approximately 80% of the wells, the medium was replaced with 2 ml of serum-free medium, inhibitor LY294002 was added for pretreatment for 1 h before incubation with 5 ng/ml TGF-β1, 20 ng/ml bFGF or 20 µg/ml bleomycin as stated above for 48 h. Then, cells of each group were washed three times with ice-cold phosphate buffer solution (PBS) and lysed in cell lysis buffer of total protein extraction kit (KeyGENBioTECH, China), following the manufacturer’s instructions, and total protein was obtained for Western blotting. Equal amounts of protein samples (30 μg) were separated on 10% sodium dodecyl sulfate (SDS)-polyacrylamide gels and electrophoretically transferred to PVDF membranes. Following blocking with 5% nonfat milk at room temperature for 2 h, membranes were incubated with the primary antibody at the appropriate dilution (ESRP1 1:800, E-cadherin1:1500, Vimentin 1:2500, α-SMA 1:1000, β-actin 1:3500) overnight at 4°C and then incubated with a horseradish peroxidase-conjugated secondary antibody (1:10,000) for 2 h at room temperature. Specific immune complexes were detected using Immobion™ Western Chemiluminescent HRP Substrate (Millipore, U.S.A.). The band density was also quantified using (Media Cybemetics Inc., Silver Spring, MA, U.S.A.). The optical density of each protein was normalized against β-actin.

### Immunofluorescence assay

A549 cells were seeded in 24-well plates, and the medium was replaced with 1 ml of serum-free medium. The inhibitor LY294002 was added for pretreatment for 1 h before incubation with 5 ng/ml TGF-β1, 20 ng/ml bFGF or 20 µg/ml bleomycin for 48 h. Cells were washed three times with PBS, fixed with 4% paraformaldehyde for 20–30 min and permeabilized with 0.5% Triton X-100 for 10 min. After blocking with goat serum for 2 h at room temperature, cells were incubated with antibodies against E-cadherin (1:100 dilution) and Vimentin (1:200 dilution) at 4°C overnight. Then, dishes were washed three times with PBS and incubated with FITC or Cy3 secondary antibodies (1:300 dilution) for 1 h at room temperature. Nuclei were stained with DAPI (10 mg/ml) for 10 min. Samples were examined with an Olympus BX43 microscope to analyze the expression of E-cadherin and Vimentin.

### Statistical analysis

All the values are expressed as the means±SD (standard deviation) of three independent experiments. Comparisons between two groups were performed using Student’s *t*-test or multiple groups by one-way ANOVA followed by post-hoc analysis. Statistical analyses were performed with SPSS software version 23 (IBM.USA). *P*-values<0.05 were considered statistically significant. Data statistics and cylindrical chart were implemented in Graph Pad Prism6 (Graph Pad Software Inc., La Jolla, CA).

## Results

### Both bFGF and TGF-β1 were up-regulated in bleomycin-induced pulmonary fibrosis

The Kunming mice were administered 6 mg/kg bleomycin, and 4 weeks later, the mice were killed, and lung tissues were collected for histology or immunohistochemistry analysis. H&E (Figure 1A) and Masson’s trichrome staining (in which muscle fiber was stained for red color and collagen fiber was stained for blue color, respectively) (Figure 1B) were used to assess pulmonary fibrosis. Compared with the control mice, bleomycin treatment induced significant changes in alveolar structure, resulting in thicker alveolar septal space and narrower alveolar space in bleomycin-treated mice, and the overall architecture of tissues was markedly distorted. Additionally, increased collagen deposition was also observed in bleomycin-treated mice. These data suggest that BML treatment induced pulmonary fibrosis in mice.

**Figure 1:** Both bFGF and TGF-β1 are up-regulated in bleomycin-induced pulmonary fibrosis Mice were treated with inhaled bleomycin or saline at 6 mg/kg for 4 weeks, the lung tissues were processed, and (**A**) pulmonary fibrosis was determined by hematoxylin–eosin (H&E) staining (20× and 40×, respectively). (**B**) Collagen was detected by Masson’s trichrome staining (20× and 40×, respectively). (**C,D**) The levels of bFGF and TGF-β1 in the lung tissues of bleomycin-induced pulmonary fibrosis were examined by immunohistochemistry (20× and 40×, respectively). (**E,F**) bFGF and TGF-β1 levels in bleomycin-treated A549 culture supernatants were detected using an ELISA kit; *P < 0.05, **P < 0.01.

In addition, significantly increased expression of bFGF and TGF-β1 was detected by IHC in the lung tissue of bleomycin-treated mice compared with control mice (Figure 1C,D). Consistent with the *in vivo* results, we also detected high concentrations of TGF-β1 and bFGF in the conditioned media from the bleomycin-treated A549 cells compared with the control cells (Figure 1E,F). These findings suggest that TGF-β1 and bFGF may be involved in bleomycin-induced lung fibrosis.

### Both bFGF and TGF-β1 promoted EMT in A549 cells

Previous studies showed that bFGF and TGF-β1 play crucial roles in EMT and fibrosis [27,28]. Consistent with previous studies, our data also show that the cell morphology of bFGF- or TGF-β1-treated A549 cells was more scattered, slender and fibroblast-like (Figure 2A). Further, to assess EMT in bFGF- or TGF-β1-treated 549 cells, related markers were detected both through Western blotting and immunofluorescence assays. In the presence of bFGF or TGF-β1, we observed up-regulated protein expression of Vimentin and down-regulated protein expression of E-cadherin in bFGF- or TGF-β1-treated A549 cells compared with their control group. We also observed increased protein expression of α-SMA by bFGF or TGF-β1 treatment (Figure 2B). α-SMA belongs to the actin family members, which are expressed largely in EMT or cancer cells [29]. Moreover, the effects of fibro genic stimuli were investigated by immunofluorescence assay in A549 cells to evaluate the occurrence of EMT. E-cadherin and Vimentin were marked in A549 cells that were exposed to 20 ng/ml bFGF and 5 ng/ml TGF-β1 for 48 h, as evidenced by the dramatic increase in Vimentin expression (red signal) and decrease in E-cadherin expression (green signal) (Figure 2C).

**Figure 2:** Both bFGF and TGF-β1 promote epithelial–mesenchymal transition in A549 cells (**A**) Cell morphology of CK and bFGF or TGF-β1-treated A549 cells. (**B**) The relative protein levels of E-cadherin, Vimentin and α-SMA were detected in A549 cells incubated with 20 ng/ml bFGF or 5 ng/ml TGF-β1 for 48 h. (**C**) E-cadherin (green signal) and Vimentin (red signal) of the CK, bFGF and TGF-β1-treated groups were examined by immunofluorescence; *P < 0.05, **P < 0.01.

### The expression of ESRP1 was down-regulated by BML, TGF-β1 and bFGF

Previous reports have shown that TGF-β drives EMT by down-regulating ESRP1 [30]. Thus, we investigated the effects of ESRP in BML-induced lung fibrosis and EMT. As shown in Figure 3, ESRP1 expression was significantly decreased in the lung tissues of BLM-treated mice compared with control mice lung tissues (Figure 3A). *In vitro* results also show that BLM treatment dramatically inhibited ESRP1 expression in A549 cells (Figure 3B). In addition, bFGF and TGF-β1 down-regulated ESRP1 expression at both mRNA (Figure 3C) and protein (Figure 3D) levels. These findings suggest that ESRP1 may be involved in BLM-induced lung fibrosis.

**Figure 3:** The expression of ESRP1 was down-regulated by BML, TGF-β1 and bFGF (**A**) ESRP1 was examined by immunohistochemistry (20× and 40×, respectively). (**B**) The A549 cells were incubated with 20 µg/ml bleomycin in serum-free medium for 48 h, and then the RNA was collected for quantitative real-time PCR to evaluate mRNA levels of *ESRP1*. (**C**) Relative mRNA levels of *ESRP1* in A549 cells were down-regulated after incubation with 20 ng/ml bFGF or 5 ng/ml TGF-β1 for 48 h. The data were normalized to the CK group. (**D**) The relative protein level of ESRP1 in A549 cells was down-regulated after incubation with 20 ng/ml bFGF or 5 ng/ml TGF-β1 for 48 h; *P < 0.05, **P < 0.01.

### ESRP1 knockdown triggered EMT in A549 cells

Here, we investigated whether ESRP1 is involved in EMT. As expected, our results show that silencing ESRP1 (Figure 4A,B) caused more scattered cell density and more fibroblast-like cells (Figure 4C). Immunohistochemistry was implemented to identify E-cadherin and Vimentin in each group. Green-marked E-cadherin surrounded the nucleus, and some Vimentin was observed in the NC group, while considerable Vimentin, which is marked with red, was observed in siESRP1-002 and shows some E-cadherin (Figure 4D). In the qRT-PCR results, the mesenchymal marker *Vimentin* in the siESRP1 group demonstrated different levels of up-regulation compared with the NC group, while the epithelial marker *E-cadherin* was down-regulated with siESRP1, all of which achieved significant differences (Figure 4E). Identical phenomena appeared in the Western blot results. Relative protein expression of mesenchymal markers Vimentin and α-SMA in the siESRP1 groups indicated great increases with extremely significant differences (*P* < 0.01). However, the expression of E-cadherin was significantly reduced (*P* < 0.01) in the siESRP1 knockdown cells (Figure 4F). These results illustrate that ESRP1 plays a vital role in EMT.

**Figure 4:** ESRP1 knockdown triggered epithelial–mesenchymal transition in A549 cells (**A**) Relative mRNA expression of *ESRP1* in A549 cells transfected with nontargeting signal silence control siRNA (NC) or ESRP1 siRNA (siESRP1-001, siESRP1-002, siESRP1-003). (**B**) Western blot analysis of ESRP1 in A549 cells transfected with NC siRNA or ESRP1 siRNAs. (**C**) Cell morphology of NC and siESRP1-002 cells was revealed (10×). (**D**) Immunohistochemistry was implemented to observe the E-cadherin (green) and Vimentin (red) in each group (20×). (**E**) Quantitative real-time PCR of the mesenchymal marker *Vimentin* and epithelial marker *E-cadherin* were detected in the NC and siESRP1-002 groups. (**F**) Western blot analysis of Vimentin, α-SMA and E-cadherin in the NC and siESRP1-002 groups; *P < 0.05, **P < 0.01.

### Bleomycin induced EMT partly through bFGF/PI3K/Akt/ESRP1 signaling in A549 cells

In previous studies, we demonstrated that bleomycin induces EMT partly through activating TGF-β/Smad/ESRP1 signaling [17,30]. However, the mechanism of bFGF in bleomycin-induced EMT is not clear. The PI3K/Akt pathway can be activated by bFGF and plays an important role in lung fibrosis and EMT [31,32]. Thus, we investigated the effects of bFGF-activated PI3K/Akt signaling in bleomycin-induced EMT. First, we identified significantly increased Akt phosphorylation by bFGF but not by TGF-β1in A549 cells (Figure 5A), suggesting bleomycin-induced Akt signaling activation mainly through bFGF. Next, we investigated the effects of PI3K-Akt/ESRP1 signaling on bleomycin-induced EMT. Our results showed that inhibition of PI3K/Akt signaling using the PI3K inhibitor LY294002 (Figure 5B) significantly inhibited bleomycin-induced morphological changes in A549 cells (Figure 5C); however, the effects of the PI3K inhibitor LY294002 were inhibited by ESRP1 silencing (Figure 5C,D). Consistent with cell morphology changes, treatment with the PI3K inhibitor LY294002 inhibited bleomycin-induced down-regulation of E-cadherin and up-regulation of α-SMA and Vimentin inA549 cells, and the effects of LY294002 were inhibited by silencing ESRP1 (Figure 5E). Furthermore, we confirmed these results using immunofluorescence and observed similar results as before (Figure 5F). Taken together, these findings suggest that bFGF stimulates EMT through PI3K/Akt/ESRP1 signaling in bleomycin-induced EMT.

**Figure 5:** Bleomycin induced EMT partly through bFGF/PI3K/Akt/ESRP1 signaling in A549 cells (**A**) The phosphorylation of pAKT/AKT in bFGF or TGF-β1-treated A549 cells was evaluated. (**B**) The phosphorylation of pAKT/AKT in BLM-treated and ESRP1-silenced A549 cells was evaluated. (**C**) Cell morphology of the four groups (CK, BLM, BLM-LY, BLM-LY-siESRP1) was displayed. (**D**) The relative mRNA level of ESRP1 in A549 cells was down-regulated after incubation with 20 µg/ml bleomycin and siESRP1, while the expression was increased after treatment with the PI3K inhibitor LY294002. (**E**) Western blot analysis of Vimentin, α-SMA and E-cadherin in the control and other three experimental groups (BLM, BLM-LY, BLM-LY-siESRP1). (**F**) Immunohistochemistry was implemented for evaluating the E-cadherin (green) and Vimentin (red) in each group (20×). BLM labeled in figures indicates bleomycin, LY labeled in figures indicates the PI3K inhibitor LY294002; *P < 0.05, **P < 0.01.

## Discussion

### ESRPs are indispensable regulators of EMT and pulmonary fibrosis events

Idiopathic pulmonary fibrosis (IPF) is a chronic disease with high mortality that is characterized by a progressive lung disorder of unknown etiology. Previous studies have concluded that EMT is an indispensable process of IPF. Epithelial cells experience alterations in epithelial function, increased extracellular matrix deposition, fibroblast activation and morphological changes to mesenchymal cells. The investigation of EMT events can be traced back to the 1980s, and more mechanisms are being uncovered [25]. ESRP1 and ESRP2 were reported as master splicing regulators in EMT, involved in the transformation of epithelial FGFR-IIIb and mesenchymal FGFR-IIIc, which are two isoforms of FGFRs [33]. Genome-wide determination study show that ESRP (ESRP1 and ESRP2) participation in pathways and protein interaction networks that are likely to have important roles in EMT [9]. In fact, a report show that altered expression and splicing of ESRP1 in malignant melanoma correlates with epithelial–mesenchymal status [34]. Importantly, Jeong et al. report that overexpression of ESRP1 can inhibit EMT in ovarian cancer [35]. In addition, our previous study shows that BLM inhibited ESRP1 expression, resulting in enhanced alternative splicing of FGFR2 to the mesenchymal isoform IIIc, thereby induces EMT in the lung fibrosis [26]. Taken together, these findings suggesting that ESRP1 plays crucial role in EMT and fibrosis. However, the regulation of ESRP1 expression is not fully understood.

### Pulmonary fibrosis inducer, bleomycin, regulates ESRP by increasing TGF-β1 and bFGF expression

Among the numerous pulmonary fibrosis/EMT models, the most common and successful model is bleomycin-induced pulmonary fibrosis/EMT, both *in vivo* and *in vitro* [17,24,36]. Previous studies verified that BLM can induce EMT of A549 cells via the TGF-β1/Smad signaling pathway and can increase the expression of bFGF and TGF-β1 [28]. In our results, the BLM-induced pulmonary fibrosis model was displayed by histology and immunohistochemistry staining. Characteristics of pulmonary fibrosis, such as thicker alveolar septum, narrower alveolar space and unformed alveolar structure, were demonstrated in the lungs of BLM-treated mice (Figure 1A,B). A549 cells treated with BLM, bFGF and TGF-β1 all experienced EMT, presented as fibroblast-like cells with more scattered cell density and more slender cell morphology (Figures 2A and 5C). In the present study, we first verified the increase in bFGF and TGF-β1 in bleomycin-induced EMT and pulmonary fibrosis (Figure 1C–F). Simultaneously, the decreased expression of ESRP1 was detected in BLM-treated mice and A549 cells (Figure 3A,B). Moreover, the decreased expression of ESRP1 was also demonstrated in bFGF- and TGF-β1-treated A549 cells (Figure 3C,D). Notably, silencing ESRP1 also promoted EMT in A549 cells (Figure 4C). Therefore, we suspect that in BLM-induced EMT and regulated ESRP1, most likely by increasing TGF-β1 and bFGF expression.

### bFGF promoted EMT via PI3K/Akt signaling pathways in bleomycin-induced EMT

Studies have identified BLM-induced EMT via the TGF-β1/Smad signaling pathway [17]; however, the bFGF-PI3K/Akt signaling pathway in BLM-induced EMT has rarely been reported. Our findings suggesting that BLM treatment caused up-regulation of bFGF was involved in stimulation of lung fibrosis and EMT. Our results also supported by other research group studies. Inoue et al*.* study also show that bFGF might exert fibrogenic in the lung [37]. Notably, bFGF antisense oligonucleotide therapy shows that it can prevent the development of pulmonary fibrosis in animals [38], suggesting that bFGF stimulates lung fibrosis and it is a important target for lung fibrosis therapy. The downstream effectors of bFGF were phosphatidylinositol 3-kinase (PI3K), mitogen-activated kinases, protein kinase B (Akt) and glycogen synthase kinase 3β (AKT/GSK-3β), and PI3K/Akt and AKT/GSK-3β pathways were obviously activated in bFGF-induced EMT [16,39,40], and when PI3K/Akt was blocked, the effects of bFGF on EMT were weakened [41]. Thus, we speculated that the bFGF-PI3K/Akt signaling pathway also play an important role in BLM-induced EMT, which is classified as a non-Smad signaling pathway. This speculation was proved by the results in Figure 5. The PI3K inhibitor LY294002 was added to BLM-treated A549 cells, and the cells became less fibroblast-like and tended to appear more like normal cells (Figure 5C), suggesting that PI3K/Akt pathway is important target candidate for lung fibrosis treatment or prevention. Furthermore, the results showed a significant increase in Akt phosphorylation in bFGF-treated A549 cells but not in TGF-β1 cells (Figure 5A), indicating that bleomycin-induced PI3K/AKT signaling was activated mainly by bFGF. These results indicate that the non-Smad signaling pathway of bFGF-PI3K/Akt signaling plays a critical role in BLM-induced EMT.

## Conclusion

In summary, our findings clearly indicate that bleomycin induces overexpression of bFGF, and overexpressed bFGF promotes EMT in the lung through inhibition of ESRP1 expression by activating PI3KAkt signaling pathway. Our results establish a new mechanism of bleomycin-induced EMT and may provide an important basis for the treatment of pulmonary fibrosis and related diseases.

## Abbreviations

bFGF: basic fibroblast growth factor
BLM: bleomycin
EGF: epidermal growth factor
EMT: epithelial-to-mesenchymal transition
ESRP: epithelial splicing regulatory protein
FGF: fibroblast growth factor
FGFR: fibroblast growth factor receptor
HCC: hepatocellular carcinoma
PF: pulmonary fibrosis
PI3K: phosphatidylinositol 3 kinase
TGF-β1: transforming growth factor-β1
